# The Value of Vaginal Microbiome in Patients with Endometrial Hyperplasia

**DOI:** 10.1155/2021/4289931

**Published:** 2021-12-18

**Authors:** Hu Zhang, Qiao Feng, Zhanpeng Zhu, Haiyan Dai, Hua Hu

**Affiliations:** ^1^Department of Gynecology and Obstetrics, Shanghai Pudong Hospital, Fudan University Pudong Medical Center, 2800 Gongwei Road, Pudong, Shanghai 201399, China; ^2^Departement of Gynecology and Obstetrics, The Second Affiliated Hospital, Third Military Medical University (Army Medical University), 183 Xinqiao Street, Shapingba, Chongqing 400037, China

## Abstract

**Objective:**

To investigate the profiles of the vaginal microbiome in patients with endometrial hyperplasia and to explore the potential value of vaginal microbiome in the diagnosis of endometrial hyperplasia. *Materials/Methods*. 26 patients suffering from abnormal uterine bleeding (AUB) with thickened endometrium revealed by transvaginal ultrasonography were enrolled. Based on pathology, 12 patients with endometrial hyperplasia were classified as the Veh group and 14 patients with proliferative endometrium were classified as the Vne group. The vaginal samples were collected for the presence of microbial DNA by high-throughput next-generation sequencing of the 16S rRNA gene. The *α*-diversity and *ß*-diversity of vaginal microbiome were analyzed and compared between bacterial populations. The ROC curve was made to evaluate the feasibility of flora as a biomarker.

**Results:**

The diversity of vaginal microbiome in the Veh group was significantly lower than that in the Vne group (*P* < 0.05). *Lactobacillus* was the most represented genus in the Veh group. The study's *t*-test between the two groups showed that *Lactobacillus* has the only significant difference in the abundance of the first 15 genera (*P* < 0.01). ROC analysis of the abundance of *Lactobacillus* showed that the area of AUC was 0.83, the sensitivity was 93.00%, and the specificity was 75.00%.

**Conclusion:**

The study offers insight into the nature of the vaginal microbiome and suggests that surveying the vaginal microbiota might be useful for detection of endometrial hyperplasia.

## 1. Introduction

Endometrial hyperplasia (EH) is a common gynecological disease, which can progress or occur at the same time as endometrial carcinoma [1, 2]. Sensitive and accurate diagnosis of true premalignant endometrial lesions and treated appropriately are required. The evaluation should include clinical documentation and transvaginal ultrasonography (TVS). The first two steps only evoke a clinical suspicion of endometrial hyperplasia and then obtain histopathological results through invasive procedures for the definite diagnosis. However, it is necessary to make clear that ultrasonographic measurements are less accurate in many conditions, such as obesity. For some patients, endometrial sampling is overtreatment.

Endometrial hyperplasia results from the continuous hyperestrogenic effect and lack of progesterone protection [3, 4]. It has reported that there is a significant correlation between estrogen and vaginal microbiome by University of Arkansas for Medical Sciences' researcher [5]. Unfortunately, few studies on vaginal microbiome in patients with EH, especially the characteristics of EH vaginal flora, are still unclear. The purpose of this study is to explore the character and to access the value of vaginal microecology in patients with endometrial hyperplasia.

## 2. Materials and Statistical Analysis

### 2.1. Methods

This study included 26 patients who were afflicted with “abnormal uterine bleeding” and “endometrial thickness” revealed by TVS in the Department of Obstetrics and Gynecology of Shanghai Pudong Hospital from September 2017 to January 2020. The pathological results were obtained by diagnostic curettage or hysteroscopy, including 14 patients with proliferative endometrium as the Vne group and 12 patients with endometrial hyperplasia as the Veh group (simple hyperplasia, *n* = 4; complex hyperplasia without atypia, *n* = 3; and complex atypical hyperplasia, *n* = 5). The pathologic diagnosis for all patients was performed by two experienced gynecologic pathologists. The Ethical Committee of Shanghai Pudong Hospital approved the study protocol, and informed consent of all individual participants was obtained in the study. The inclusion criteria were as follows: (1) age between 30 and 65 with abnormal uterine bleeding; (2) no recorded recent use of abnormal vaginal discharge, vaginal medications, and antibiotics, hormones, no cervical treatment within a week; (3) no douching and no sexual activity within 48 h; (5) endometrial thickness in postmenopausal patients >5 mm and in nonpostmenopausal patients >10 mm after 3 days of menstruation. Exclusion criteria: (1) pregnant or lactating women; (2) vaginal inflammatory diseases; (3) cancer, endocrine, or autoimmune disease. Clinical data were collected through the inpatient medical record system. Detailed clinical data are given in Table 1.

### 2.2. Samples Collection

All vaginal samples were collected before vaginal lavage, disinfection, and operation from the upper third vagina. The sterilized cotton swabs lightly rotated on the vagina for about 10–15 s. 3 swabs of each subject were performed with a sterile test tube on ice and immediately placed in a transfer container with ice, stored in refrigerator (−80°C) within 1 h, and transported in dry ice to Majorbio Company (Majorbio, Shanghai, China).

### 2.3. DNA Extraction and PCR Amplification

Microbial DNA was extracted from vaginal samples using the TransStart FastPfu DNA Polymerase (TransGen Biotech, Beijing, China) according to manufacturer's protocols. The final DNA concentration and purification were determined by the NanoDrop 2000 UV-vis spectrophotometer (Thermo Scientific, Wilmington, USA), and DNA quality was checked by 1% agarose gel electrophoresis. The V3-V4 hypervariable regions of the bacteria 16S rRNA gene were amplified with primers 338F (5′-ACTCCTACGGGAGGCAGCAG-3′) and 806R (5′-GGACTACHVGGGTWTCTAAT-3′) by the thermocycler PCR system (GeneAmp 9700, ABI, USA). The PCR reactions were conducted using the following program: 3 min of denaturation at 95°C, 27 cycles of 30s at 95°C, 30 s for annealing at 55°C, and 45 s for elongation at 72°C, and a final extension at 72°C for 10 min. PCR reactions were performed in triplicate: 20 *μ*L mixture containing 4 *μ*L of 5× FastPfu Buffer, 2 *μ*L of 2.5 mM dNTPs, 0.8 *μ*L of each primer (5 *μ*M), 0.4 *μ*L of FastPfu Polymerase, and 10 ng of template DNA. The resulted PCR products were extracted from a 2% agarose gel and further purified using the AxyPrep DNA Gel Extraction Kit (Axygen Biosciences, Union City, CA, USA) and quantified using QuantiFluor™-ST (Promega, USA) according to the manufacture's protocol. Purified amplicons were pooled in equimolar and paired-end sequenced (2 × 300) on an Illumina MiSeq platform (Illumina, San Diego, USA) according to the standard protocols by Majorbio BioPharm Technology Co., Ltd. (Majorbio, Shanghai, China).

### 2.4. Processing of Sequencing Data

Raw fastq files were quality-filtered by Trimmomatic and merged by FLASH with the following criteria. (i) The reads were truncated at any site receiving an average quality score <20 over a 50 bp sliding window. (ii) Sequences whose overlap being longer than 10 bp were merged according to their overlap with mismatch no more than 2 bp. (iii) Sequences of each sample were separated according to barcodes (exactly matching) and primers (allowing 2 nucleotide mismatching), and reads containing ambiguous bases were removed. Operational taxonomic units (OTUs) were clustered with 97% similarity cutoff using UPARSE (version 7.1 http://drive5.com/uparse/) with a novel “greedy” algorithm that performs chimera filtering and OTU clustering simultaneously. The taxonomy of each 16S rRNA gene sequence was analyzed by the RDP classifier algorithm (http://rdp.cme.msu.edu/) against the SILVA (SSU132) 16S rRNA database using confidence threshold of 70%.

### 2.5. Data Processing

The original image data (raw data) obtained from the second-generation sequencing is converted into sequence data by base recognition (base calling), the sequencing sequence is controlled by Trimmomatic software, spliced by FLASH software, OUT analysis is carried out by UPARSE software, taxonomic analysis of OUT representative sequence is carried out by the RDP classifier Bayesian algorithm, and OUT is compared to SILVA database by Mothur analysis flow. Annotate the species (the threshold is set to 0.7). The difference of alpha diversity between groups was tested by the Shannon algorithm and Simpson algorithm, and the species composition was analyzed by R language based on the data table in tax summary folder. The diversity of beta was analyzed by NMDS (nonmetric multidimensional scaling analysis) statistical analysis of R language, the difference of bacteria between the two groups was tested by ANOSIM values based on Bray–Curtis dissimilarity at the genus level, and sequence data were mainly analyzed using the QIIME, Mothur1.30.2, SILVA132, UPARSE 7.0.1090, USEARCH 7.0, RDP classifier, and R packages (v3.2.0). In addition, sequencing data were also analyzed using the free online Majorbio I-Sanger Cloud Platform (https://www.i-sanger.com). Then, we performed differential abundance analysis to distinguish which taxa contributed to the validated microbiome structural changes in the vaginal microbiome of the Veh group. The *P* value (*P*) < 0.05 was considered to reflect a statistically significant difference. The receiver operating characteristic (ROC) curve and area under the curve (AUC) were analyzed by R packages (v3.2.0) (R Development Core Team, Vienna, Austria).

### 2.6. Statistical Analysis

The data were statistically analyzed by SPSS version 21.0 for Windows (SPSS Inc., Chicago, IL, USA) in which the data of age, body mass index (BMI), and endometrial thickness were in accordance with normal distribution, expressed by mean ± standard deviation (means ± SD), and compared between groups by the *t*-test. The counting data of menopause, hypertension, and diabetes were expressed by percentage, the chi-square test was used for comparison between groups, and the rank-sum test was used for the number of births and abortions. The difference was statistically significant (*P* < 0.05).

## 3. Results

### 3.1. Baseline Characteristics

The age of the enrolled patients ranged from 31 to 62, with Vne patients between 38 and 62 years old (mean age:47.71 ± 6.78 years, mean ± standard error), Veh between 31 and 57 years old (mean age:45.17 ± 6.21 years, mean ± standard error). The Veh group consisted of 4 simple hyperplasias, 3 complex hyperplasias without atypia, and 5 complex atypical hyperplasias; 14 proliferative endometriums were sorted as the Vne group. The patients` clinical data are listed in Table 1. The mean age, the case of menopause, hypertension and diabetes, BMI index, times of gravida and parity, Histotype and endometrial thickness between the Vne group and the Veh group were not statistically significant.

### 3.2. Sequencing Information

In this experiment, a total of 1,337,846 high quality gene sequences (31,582–72,918) were obtained, with an average of 51,455 reads per sample. A total of 1,250 OTUs and 712 OTUs were detected in the Vne and Veh groups, respectively. Both groups shared 453 OTUs. A total of 516 genera of bacteria were detected in all vaginal samples, including 305 genera in the Vne group and 279 genera in the Veh group. Both groups shared 68 genera.

### 3.3. Difference of Bacterial Community between the Two Groups

We first compared the overall microbiota structure between disease states by analyzing the *α*-diversity and *ß*-diversity. The *α*-diversity (Shannon, Simpson, and Heip indices of the vaginal microbiota in OTU and genus level) in the Veh group was significantly lower (*P* < 0.05) than that of the Vne group (Tables 2 and 3). Significant differences were also found in *ß*-diversity based on the Bray–Curtis though NMDS was based on genus level (*P*=0.008) between the Vne and Veh groups (Figure 1).

*P* values are reported combining the evidence across the Bray–Curtis, ANOSIM, and multiple displacement amplification: 999(stress: 0.138, *R* = 0.214, *P*=0.008). NMDS is the evaluation of the rank information of the distance value. NMDS1 and NMDS2 axes do not have the weight of meaning. The overall dimensionality reduction effect of NMDS is judged by the stress value.

Our data showed that the vaginal microbial community diversity and community evenness were significantly lower in the Veh group than in the Vne group in OTU and genus level.

We second conducted flora structure constituting ratio analysis. The species composition of phylum in the Vne group from high to low is Firmicutes: 41.01%, Actinobacteria: 33.34%, Bacteroides: 15.59%, and other bacteria accounted for 10.05%. The phylum of bacteria in the Veh group is the same as that in the Vne group, but the constituent ratio is different. Among them, the proportion of Firmicutes increased to 64.92%, Actinobacteria decreased to 22.63%, Bacteroidetes decreased to 6.34%, and other bacteria accounted for 12.45% (Figure 2).

At the level of bacteria genus, the highest vaginal bioabundances in the Vne group were *Gardnerella*, *Prevotella*, *Atopobium*, and *Lactobacillus*, and their percentages were 17.06%, 14.07%, 13.59%, and 11.29%, respectively. In the Veh group, 58.76% of *Lactobacillus*, 21.61% of *Gardnerella*, and 6.05% of *Prevotella* were the highest (Figure 2).

To get more insight into the characteristics of the patient's microbiome, we conducted a differential analysis of microbial abundance. In class, order, family, and genus levels, the Bacilli, Lactobacillales, Lactobacillaceae, and *Lactobacillus* were significantly higher in the Veh group than in the Vne group. After the overall microbiome assessment, only *Lactobacillus* has statistically significant different abundances of the top 15 bacterial genera. The abundance of *Lactobacillus* in the Veh group was significantly higher than those in the Vne group (*P* < 0.05) (Figure 3).

Through the ROC prediction analysis of the patients with thickened endometrium with the abundance of *Lactobacillus* by R packages (v3.2.0), the ROC curve was obtained, which showed that the AUC area was 0.83, the sensitivity was 93.00%, and the specificity was 75.00%, as shown in Figure 4.

## 4. Discussion

Here, we present a pilot high-throughput microbiome assessment of the female vaginal of patients diagnosed with a benign uterine condition (thickened endometrium). The dominant taxa in the vaginal microbiome were *Lactobacillus*, *Gardnerella*, and *Prevotella*, consistent with current vaginal microbiome literature [6]. *Gardnerella* was the dominant flora in the proliferative endometrium group, with uniform distribution of vaginal microorganisms and rich microbial diversity. The dominant vaginal flora of patients with endometrial hyperplasia was *Lactobacillus*, and the diversity of bacteria decreased significantly.

The patients with endometrial hyperplasia were affected by high concentration of estrogen for a long time, which caused vaginal mucosal edema and increased vaginal mucosal permeability. Estrogen promotes the growth of epidermal cells and the increase of intracellular glycogen in the upper part of the vagina, which leads to the increase of *Lactobacillus*. These bacteria ferment glycogen into glucose and finally transform into lactic acid, which maintains the low PH state of the vagina. At the same time, *Lactobacillus* inhibits the growth of other bacteria by producing H_2_O_2_, which further strengthens the dominant position of *Lactobacillus*, resulting in a decrease in the diversity of bacteria [7]. In the past, we found only one study about the distribution of vaginal microorganisms in patients with endometrial hyperplasia. However, in contrast with our data, it reported that the lower genital tract microbiome structure of the hyperplasia cohort was not distinguishable from the benign cohort [8]. The vaginal microbiome of these hyperplasia patients resembled a benign microbiome signature. The discrepancy may be caused by the difference of sample sources, sample quantity, race, age, and menopausal years [9].

Our results indicate that endometrium hyperplasia can be distinguished by the vaginal microbial community diversity and community evenness. The vaginal *α*-diversity of the Veh group was significantly lower than the Vne group.

Through ROC curve analysis, we found that the abundance of *Lactobacillus* can be used as a landmark microorganism for differential diagnosis of endometrial thickening, with a sensitivity of 93.00% and a specificity of 75.00%. Our results suggest that the detection of *Lactobacillus* in the vagina is associated with the presence of endometrial hyperplasia. Since we do not have healthy asymptomatic patients in this research, we cannot assess whether this correlation exists or does it indicate illness status. The causal relationship needs further study. There are few reports on the differential diagnosis of patients by microbiome identification [10]. It has an important value for avoiding medical overuse such as diagnostic curettage, hysteroscopy, and other invasive procedures and economic burden.

However, this study also has some defects. On the one hand, the small sample size of single center, and on the other hand, there are no confounding factors such as vaginal microbial PH value, menstrual interval, bleeding interval, estrogen level, menopausal time, uterine leiomyoma, adenomyosis, delivery mode, and so on. In addition, due to the heterogeneity and dynamics of vaginal microecology, long-term follow-up and microbial samples in different periods still need to be further studied.

## 5. Conclusions

We found a distinct microbiome signature in patients with endometrial hyperplasia. We have shown that the detection of *Lactobacillus* in the gynecologic tract was associated with the presence of endometrial hyperplasia in our study population. These findings provide important insights into the etiology or manifestation of the disease with broad implications for biomarker development in the early detection of and screening for endometrial hyperplasia by noninvasive methods.

## Figures and Tables

**Figure 1:** *ß*-Diversity measures were compared through NMDS on the genus level.

**Figure 2:** Comparison flora structure constitution in different levels. (a) Community analysis pie plot on phylum level in the Vne group. (b) Community analysis pie plot on phylum level in the Veh group. (c) Community analysis pie plot on genus level in the Vne group. (d) Community analysis pie plot on genus level in the Vne group.

**Figure 3:** Two groups of the abundance *t*-test before 15 kinds of species diversity; only *Lactobacillus* had differences between them, *P*=0.0017.

**Figure 4:** ROC curve for *Lactobacillus* presence in the vaginal tract between disease status (proliferative endometrium vs. endometrial hyperplasia).

**Table 1:** Baseline characteristics.

Variables	Vne (*n* = 14)	Veh (*n* = 12)	*P* value
Age (mean ± SD)	47.71 ± 6.78	45.17 ± 6.21	0.33
Postmenopause (%)	4 (28.57)	3 (25.00)	1
Hypertension (%)	3 (21.43)	2 (16.67)	1
Diabetes (%)	1 (7.14)	2 (16.67)	0.58
BMI (mean ± SD)	23.95 ± 4.85	26.74 ± 4.56	0.15
Gravida, range	22 (1, 3)	15 (0, 2)	0.26
Parity, range	17 (0, 2)	5 (0, 5)	0.051
Endometrial thickness (mm)	10.91 ± 5.19	13.40 ± 6.36	0.28
Histotype (%)			
Simple hyperplasia	—	4 (33.33)	
Complex hyperplasia without atypia	—	3 (25.00)	
Complex atypical hyperplasia	—	5 (41.67)	
Proliferative endometrium	14 (100)	—	

**Table 2:** *α*-diversity comparison between Vne and Veh in OTU level.

Estimators	Veh, mean	Veh, SD	Vne, mean	Vne, SD	*P* value	*Q* value
Shannon	0.751	0.76	1.649	0.958	0.015	0.041
Simpson	0.698	0.293	0.367	0.292	0.008	0.041
Heip	0.015	0.016	0.046	0.037	0.013	0.041

**Table 3:** *α*-diversity comparison between between Vne and Veh in genus level.

Estimators	Veh, mean	Veh, SD	Vne, mean	Vne, SD	*P* value	*Q* value
Shannon	0.620	0.655	1.444	0.826	0.010	0.027
Simpson	0.731	0.284	0.385	0.282	0.005	0.027
Heip	0.019	0.022	0.066	0.051	0.007	0.027

## Data Availability

The simulation experiment data used to support the findings of this study are available from the corresponding author upon request.

## References

[1] Siegel R. L., Miller K. D., Fuchs H. E., Jemal A. (2021). Cancer statistics, 2021. *CA: A Cancer Journal for Clinicians*.

[2] Travaglino A., Raffone A., Saccone G. (2019). Endometrial hyperplasia and the risk of coexistent cancer: WHO versus EIN criteria. *Histopathology*.

[3] Shang Y. (2006). Molecular mechanisms of oestrogen and SERMs in endometrial carcinogenesis. *Nature Reviews Cancer*.

[4] Hecht J. L., Mutter G. L. (2006). Molecular and pathologic aspects of endometrial carcinogenesis. *Journal of Clinical Oncology*.

[5] Mallinger W. D., Quick C. M. (2019). Benign and premalignant lesions of the endometrium. *Surgical Pathology Clinics*.

[6] Brotman R. M., Shardell M. D., Gajer P. (2014). Association between the vaginal microbiota, menopause status, and signs of vulvovaginal atrophy. *Menopause*.

[7] Tachedjian G., Aldunate M., Bradshaw C. S., Cone R. A. (2017). The role of lactic acid production by probiotic Lactobacillus species in vaginal health. *Research in Microbiology*.

[8] Walther-António M. R. S., Chen J., Multinu F. (2016). Potential contribution of the uterine microbiome in the development of endometrial cancer. *Genome Medicine*.

[9] Moosa Y., Kwon D., de Oliveira T., Wong E. B. (2020). Determinants of vaginal microbiota composition. *Frontiers in Cellular and Infection Microbiology*.

[10] Chen Y.-J., Wu H., Wu S.-D. (2018). Parasutterella, in association with irritable bowel syndrome and intestinal chronic inflammation. *Journal of Gastroenterology and Hepatology*.

